This article has been retracted.

# Analysis of risk factors related to the re-fracture of adjacent vertebral body after PKP

**DOI:** 10.1186/s40001-021-00592-w

**Published:** 2021-10-30

**Authors:** Shen-Yun Fang, Ji-Lin Dai, Ji-Kang Min, Wei-Li Zhang

**Affiliations:** 1 Orthopedics Department, The First People Hospital of Huzhou, The First People’s Hospital Affiliated to Huzhou Normal University, Huzhou, 313000 China; 2 Ophthalmology Department, The First People Hospital of Huzhou, The First People’s Hospital Affiliated to Huzhou Normal University, Huzhou, 313000 China

**Keywords:** Vertebroplasty, Vertebral compression fracture, Re-fracture, Spinal degenerative scoliosis, Osteoporosis, Risk factors

## Abstract

**Background:**

This study aims to investigate the risk factors of vertebral re-fracture after percutaneous kyphoplasty (PKP) for osteoporosis vertebral compression fracture (OVCF), and to provide reference for clinical prevention.

**Material and methods:**

A retrospective analysis was performed on 228 OVCF patients admitted on November 6, 2013, solstice, December 14, 2018, which met the inclusion criteria. There were 35 males and 193 females, with a male-to-female ratio of 3:20, and an age of 61–89 years. All patients were treated with PKP surgery with complete clinical data, and the rate of re-fracture was calculated according to whether re-fracture occurred after surgery, divided into the re-fracture group (24 cases) and the non-refracture group (204 cases). May be associated with subsequent fracture factors (gender, age, number of surgical segment vertebral body, whether with degenerative scoliosis, whether to fight osteoporosis) into a single-factor research, then the single-factor analysis was statistically significant risk factors for multiple logistic regression analysis, further defined after PKP holds the vertebral body fracture independent risk factors. Survival analysis was performed using the time of vertebral re-fracture after PKP as the end time of follow-up, the occurrence of re-fracture after PKP as the endpoint event, and the presence or absence of degenerative lateral curvature as a variable factor.

**Results:**

All 228 vertebroplasty patients were followed up for a period of 1.8 to 63.6 months. The mean follow-up time was (28.8 ± 15.6) months, and the re-fracture rate was 10.5%. There were statistically significant differences between the re-fracture group and the non-refracture group in age, number of operative vertebral bodies, whether there was a combination of degenerative scoliosis and whether there was anti-osteoporosis treatment (*P* < 0.05). The results of univariate logistic regression analysis after excluding the mutual influence of various factors showed that the number of vertebral bodies and the group with lateral curvature might be the risk factors for PKP re-fracture after surgery. The above possible risk factors were included in multiple logistic regression analysis to show whether there were independent risk factors for scoliosis and vertebral re-fracture. Survival analysis showed that the mean survival time was 42.1 months, the *P* value was 0.00, and the mean 95% confidence interval was (34.4–49.7 months), indicating that the combination of degenerative lateral bending might be related to the occurrence of re-fracture.

**Conclusions:**

Combined scoliosis is an independent risk factor for re-fracture after OVCF laminoplasty and a possible risk factor for re-fracture after surgery.

## Background

Osteoporosis (osteoporosis, OP) is a metabolic bone disease characterized by a decrease in bone tissue mass, bone microstructure destruction, and a decline in bone density and bone quality caused by a variety of factors. The morbidity rate is relatively high in the elderly, which is mainly manifested by chronic pain, restricted activities in some patients, and kyphosis in severe cases, which may even increase the mortality of patients [1, 2]. At present, the number of OP patients in China has exceeded 80 million, and its prevalence is about 6.6% of the total population, ranking first in the world, and most of the patients are elderly women over 60 years old [3]. With the aging of the social population, OP has severely affected the daily lives of middle-aged and elderly people and is listed as one of the ten most serious diseases by the WHO [4]. Osteoporotic vertebral compression fracture (OVCF) is the most common fracture type of OP [5]. The bone healing process is slow, and the patient's quality of life is low during the period, which can easily lead to various complications, which not only increases the cause. The risk of disability and mortality also brings a heavy financial burden to the patient's family [6]. According to the literature [7], OVCF has gradually become a common type of fracture in the elderly, accounting for about 45% of osteoporotic fractures.

The current treatment methods of OVCF mainly include conservative non-surgical treatment and surgical treatment; among them, surgical treatment is divided into two methods: open surgery and minimally invasive surgery. Conservative non-surgical treatment is mainly based on analgesia, bed rest, brace fixation, and physical therapy, but it cannot effectively improve kyphosis, and patients often have long-term low back pain. The purpose of OVCF surgical treatment is to shorten the time that patients stay in bed, reduce complications, reduce mortality, and improve the quality of life of patients. At present, open spinal surgery is mostly applied to patients with nerve root symptoms and spinal cord injury. However, anesthesia and surgical risks must be strictly evaluated before surgery. At the same time, severe osteoporosis may cause the screws to loosen and fall off. In 1987, Dr. Galibert used percutaneous vertebroplasty (PVP) to treat vertebral hemangioma for the first time; by the 1990s, American doctor Mark Reiley designed percutaneous kyphoplasty based on PVP, PKP), and then PVP/PKP gradually applied to the treatment of painful OVCF without spinal cord injury and nerve root symptoms, and developed into the most commonly used minimally invasive surgery for the treatment of OVCF. PVP and PKP are currently more mature minimally invasive surgery for the treatment of elderly OVCF. The more conservative treatment can quickly relieve the pain symptoms of patients, improve the stability of the vertebral body, reduce the time of lying in bed, and enable patients to resume normal activities early. They have been widely used in clinical practice [8].

Recurring vertebral body fractures after PVP can be divided into surgical vertebral body re-fractures and non-surgical vertebral body fractures. In recent years, with the increase in patients undergoing PVP and PKP surgery, there have been reports that recurring vertebral fractures after bone cement vertebral enhancement and incidence is high; Lee et al. [9] reported 402 cases of PVP treatment. OVCF patients were followed up for an average of 4.8 years, during which 120 patients had vertebral fractures again, with an incidence rate of 29.8°%; 72 patients (17.9%) had adjacent segmental vertebral fractures. Yu et al. [10] The incidence of postoperative re-fracture in the clinical studies included in the Meta-analysis was 3.21%–63%, and the cumulative incidence was 10.3%; therefore, some scholars inferred that this may be due to the filling of bone cement leading to spinal biology. However, the study by Staples et al. [11] found that patients with conservative non-surgical treatment and patients who received PVP surgery did not find a significant increase in the risk of recurring vertebral fractures during the 2-year follow-up period. Therefore, some reports speculate that recurring vertebral fractures may be the result of the development of OP. However, the current incidence of recurring vertebral fractures after PVP and related risk factors and biomechanical mechanisms have not been definitively concluded. The potential risks are still unclear. Although some articles have reported some possible risk factors, they are inconsistent or incomplete. This study analyzed the risk factors related to re-fracture after PKP operation to provide a basis for further prevention of vertebral body re-fracture after PKP operation and to guide clinical practice.

## Material and methods

### General information

We selected 228 OVCF patients who underwent PKP surgery in our hospital from November 6, 2013 to December 14, 2018. The patients were divided into a re-fractured group and a non-refractured group, including 31 males and 197 females, aged 51–91 years, with an average of (69.7 ± 7.03) years (Table 1). The fractured vertebrae included in this study included 179 cases of single vertebrae, 43 cases of two vertebrae, and 6 cases of 3 vertebrae. They were divided into re-fracture group and non-refracture group according to whether they were re-fractured after the operation. Among the 24 patients with re-fractures, 8 were in the T12–L1 segment, 6 were in the T11–T12 segment, 2 were in the L2–L1 segment, 1 was in the T10–T11 segment, 1 was in the L2–L3 segment, and T12–T9. There was 1 case in the segment, 1 case in T8–T12, 1 case in L1–L3, 1 case in L1–T11, 1 case in T12–L3, and 1 case in T12–L2. Among them, there were 17 cases of fracture with scoliosis and 7 cases of no scoliosis, but all had degenerative changes.

**Table 1:** Comparison of basic characteristics between patients with re-fracture and non-fracture

	Sex (male/female)	Age (year)	Height (m)	Weight (kg)	BMI kg/m^2^
Re-fractured group (n = 24)	4/25	75.3 ± 7.3	1.66 ± 0.08	58.73 ± 9.74	23.25 ± 4.68
Non-refractured group(n = 204)	27/172	69.0 ± 6.7	1.67 ± 0.07	60.32 ± 10.25	24.26 ± 4.55
*z*^2^ value	0.041	1.626	−1.71	−0.689	-0.883
*P* value	0.795	0.058	0.084	0.536	0.436

### Inclusion and exclusion criteria

Inclusion criteria: ① there was a certain degree of back pain before surgery, often accompanied by an inability to turn over, or a sense of weakness to get up. Local spinous process withholding tenderness; ② preoperative X-ray, CT, and MRI examinations confirmed that the vertebral compression fracture is fresh, that is, the T1 signal is low, T2 signal is a high signal or slightly high signal on MRI, and the above symptoms are combined at the same time It can be diagnosed; ③ the lumbar spine bone density measured by dual-energy X-ray bone density meter or QCT, T value < −2.5SD or less than 80 mg/dl, combined with fractures and low-energy injury, can be diagnosed as OVCF. Exclusion criteria: ① pathological fractures caused by spinal infection or tumor; ② vertebral fractures caused by high-energy injury; ③ patients with mental illness such as depression.

### Evaluation method

Judgment of risk factors: (1) basic information: collect the following factors through the HIS medical records and imaging system of the Information Department: ① gender, age; ② surgical segment; ③ number of vertebrae in operation; ④ whether it is combined with degenerative scoliosis, according to Cobb angle size, according to coronal position > 10. Defined as degenerative scoliosis of the spine; ⑤ whether it is anti-osteoporosis, postoperative anti-osteoporosis treatment (calcitonin injection, 50U, intramuscular injection, QD + calcium + vitamin D3) is given, and long-term calcium is given after discharge + Vitamin D3 maintenance treatment. Eligible patients (calculated creatinine clearance rate ≥ 35 ml/min, and no other contraindications) received an intravenous infusion of zoledronic acid needle 5 mg. The recommended course of treatment is 3 years, once a year. (2) Surgical data: in this study, PKP operations were performed with a bilateral puncture, bone cement was performed with polymethyl methacrylic (PMMA), and instruments were performed with Shanghai Kailitai Percutaneous Vertebral Expansion Balloon Angioplasty System, The operation time is 30–60 min.

Re-fracture determination: The relevant risk factors are included in the single-factor logistic study and the risk factors are screened out after statistical processing. Furthermore, the selected risk factors were analyzed by multivariate logistic regression to analyze the independent risk factors. After PKP, re-fracture of the vertebral body as the end of follow-up time, postoperative re-fracture as the end event, and whether combined with degenerative scoliosis as a variable factor, the life tables process in the survival analysis was carried out.

The re-fracture described in this article refers to the re-fracture that occurs in the adjacent vertebrae or adjacent vertebrae (including the fractured vertebrae with 1, 2, or 3 normal vertebrae outside the upper or lower vertebral body except the operative vertebrae after PKP). Re-fracture of the adjacent vertebrae refers to the fracture of the adjacent or adjacent vertebrae within a period of time after the initial fracture of the vertebral segment. Cobb kyphosis angle measurement method: the angle between the upper endplate of the fractured vertebral body and the vertical line of the lower endplate of the lower vertebral body is the "Cobb angle".

### Postoperative treatment and follow-up

A thoracolumbar brace must be worn to get out of bed the next day after surgery. The outpatient follow-up to take X-rays of the spine. The follow-up uniformly uses the last follow-up time as the end time of the follow-up. Follow-up by telephone follow-up, outpatient review, and other forms of follow-up. A follow-up plan should be made before follow-up (specific contents include: whether to fracture again after PKP/whether to continue taking calcium and vitamin D3, whether to infuse zoledronic acid injection/whether to perform imaging examination). Besides, for cases with re-fracture of the vertebral body, the time of second admission or outpatient diagnosis is the time of re-fracture. Specifically, minus the time of the first fracture diagnosis, and the time interval for re-fracture, that is, the end of follow-up time.

### Statistical processing

IBM SPSS Statistics 23 software was used for data statistical analysis. The Chi-square test was used for enumeration data, and the two-sided value was 0.05. Univariate logistic analysis was statistically significant, and then multiple logistic regression analysis was used to analyze the high-risk factors related to the occurrence of vertebral body re-fracture, and *P* < 0.05 was considered as statistically significant. The follow-up time is represented by "month". Survival analysis was performed on re-fractures and degenerative scoliosis of the spine.

## Results

### General information and follow-up

In this study, 24 cases of re-fracture occurred after PKP operation, accounting for 10.5%, and the ratio of male to female was 3:20. The age of the re-fracture group was 61–89 years, with an average of (75.3 ± 7.3) years, and the age of the non-refracture group 51–91 years, the average is (69.0 ± 6.7) years. The follow-up time was 1.8–63.6 months, with an average of (28.8 ± 15.6) months. 31 cases were lost to follow-up, with a lost-to-follow-up rate of 13.6%.

### Comparison of related factors

There were statistically significant differences between the two groups in age, the number of vertebrae operated, and whether degenerative scoliosis of the spine was combined (*P* < 0.05); there were no statistically significant differences in gender and anti-osteoporosis (*P* > 0.05). See Table 2.

**Table 2:** Comparison of risk factors between the re-fracture group and the non-refracture group

Risk factors	Group	Re-fractured group (case)	Non-refractured group (case)	*X*^2^ value	*P* value
Age	≤ 65 years	3	65	4.45	0.04
	> 65 years	21	139		
Number of vertebral bodies	≤ 1	7	172	38.71	0.00
	≥ 2	17	32		
Scoliosis	Complicated scoliosis	18	28	50.06	0.00
	Not complicated scoliosis	6	176		
Osteoporotic	Anti-osteoporotic	23	79	26.06	0.00
	Not anti-osteoporotic	1	125		
Sex	Male	4	31	0.00	1.00
	Female	20	173		

### Single-factor logistic regression analysis

The statistically significant risk factors were included in the univariate logistic regression analysis to exclude the mutual influence of the factors. The results showed that the number of vertebrae in operation and the group with degenerative scoliosis of the spine may be risk factors for re-fracture after PKP; see Table 3.

**Table 3:** Results of univariate logistic regression analysis

Risk factors	B	Standard error	Wald	Significance	Exp (B)	Exp(B) 95% confidence interval	
						Lower limit	Upper limit
Scoliosis	−2.128	0.647	10.82	0.001	0.119	0.034	0.423
Sex	−0.432	0.712	0.369	0.543	0.649	0.161	2.618
Age	0.041	0.040	1.093	0.296	1.042	0.964	1.126
Number of vertebral bodies	1.016	0.447	5.159	0.023	2.763	1.149	6.640
Whether anti-osteoporotic	0.279	0.534	0.273	0.601	1.321	0.464	3.761

### Multivariate logistic regression analysis

Incorporating the risk factors revealed by univariate regression analysis into the multiple logistic regression analysis showed that combined spinal degenerative scoliosis [OR = 0.111, 95% CI (0.036, 0.345), *P* = 0.00] was an independent risk factor for vertebral body re-fracture.

### Survival analysis

The life table showed that the median survival time of the two groups was, respectively, 48.98 months in the combined scoliosis group; 63.0 months in the non-combined scoliosis group. The Wilcoxon test value was 42.64 and the *P*-value was 0.00, indicating that the combined spinal degenerative scoliosis may be related to the occurrence of re-fracture; see Fig. 1. A typical case is shown in Fig. 2.

**Fig. 1:** Association between degenerative scoliosis and re-fracture. A, 78-year-old, female patient, primary diagnosis: osteoporotic L1 vertebral compression fracture (2016-11-18), lumbar degenerative scoliosis. **2a**, **b**. The X-ray film of the anterior and lateral position of the lumbar spine showed L1 vertebral compression fracture and degenerative scoliosis before the operation; **2c**, **d:** the X-ray film of the anterior and lateral position of the lumbar spine reexamined 2 months after the operation indicated that the bone cement in the L1 vertebral body was in place; **2e**, **2f** PKP was performed again 6 months after the operation due to compression fracture of the T12 vertebral body, and the X-ray film of the anterior and lateral position of the lumbar spine reexamined that the bone cement was well distributed; **2g**,** h** PKP was performed again in the first half of the year because of compression fracture of thoracic vertebrae 10 and 11. After the operation, the X-ray plain film of lumbar vertebrae showed that bone cement was in place

**Fig. 2:** Survival analysis suggests that combined spinal degenerative scoliosis may be associated with the occurrence of re-fracture

## Discussion

OP is a bone metabolism disease, which is mainly manifested by bone mineral density (BMD) and bone quality decline, which eventually leads to a decrease in the strength of the body's bones and an increase in bone fragility; it is irreversible in the human aging process, so it is easy to cause fractures in daily activities or minor trauma happened [12]. According to the results of the 2013 census, the number of OP patients in my country may reach 212 million by 2050. With the aging of the social population, the incidence of OP is increasing year by year, and now it has leaped to third place in chronic diseases, closely following the cardiovascular system. After illness and diabetes [13], pain, kyphosis, and fracture are the most typical clinical manifestations of OP; among them, pain is the most common clinical symptom of OP, mainly in low back pain; because the vertebral body is mostly composed of cancellous bone, it is in the place where the stress is concentrated in the spine. It is prone to compression and deformation, which will eventually lead to kyphosis. Fractures, as the most common and most serious complication of the degenerative OP, often occur in areas rich in cancellous bone. OVCF is the most common type of fracture, in severe osteoporosis. Under the circumstances, even minor trauma can cause vertebral compression fractures.

In the past 10 years or so, the incidence of re-fractures of adjacent vertebral bodies after PKP has been increasing. Su et al. [14] conducted a cohort study on the treatment of osteoporotic compression fractures with kyphoplasty and collected more than 100 patients. The incidence of re-fractures reached 27.8%, and 68% occurred in adjacent vertebrae. The re-fracture rate in this study was 10.5%, which was lower than reported. This may be related to the patient's failure to seek medical attention in time after surgery. There are different opinions on the reasons for re-fractures after surgery. The natural development of osteoporosis, biomechanical changes, and excessive injection of bone cement, and leakage of bone cement into the intervertebral disc are still controversial. However, with the deepening of research on recurring vertebral fractures after PVP, many scholars have found that the recurring vertebral fractures after PVP are mostly in the adjacent segments of the vertebral body, and the incidence is relatively high, which prompts everyone to focus to gather here.

The recurrence of vertebral body fractures after PVP is mainly divided into re-fracture of vertebral body after operation and non-surgical vertebral body fracture. Lee et al. [9] reported 402 cases of OVCF patients who received PVP treatment with an average follow-up of 4.8 years. During this period, 120 patients had vertebral fractures again, the incidence rate was 29.8%; 72 cases (17.9%) were adjacent segment vertebral fractures. The incidence of postoperative re-fracture in the clinical studies included in the meta-analysis by Yu et al. [10] was 3.21% to 63%, and the cumulative incidence was 10.3%. Yang et al. [15] compared and analyzed 290 cases of PVP and 270 cases of OVCF who underwent conservative treatment. They were followed up for at least 24 months on average and found that the probability of recurring vertebral fractures after surgery was 12.8%. Takahara et al. [16] also confirmed that the location of recurring vertebral body fractures after PVP seems to be more likely to occur in adjacent segments, and the time of adjacent vertebral fractures is earlier than that of non-adjacent vertebral fractures. In this study, the incidence of recurrence of vertebral fractures in selected patients was 13.8%, which was similar to the results of some of the above studies. The time to the reoccurrence of vertebral body fractures, the results of this study showed: 10 patients appeared within 3 months after surgery, 22 patients appeared within 6 months after surgery, 24 patients appeared within 1 year after surgery, respectively, accounting for 54.5%, 66.7%, 72.7%, the results show that within 1 year after PVP surgery is an important time period for recurring vertebral fractures. Reviewing the relevant literature, due to differences in inclusion criteria, follow-up years, and statistical methods, the reported incidence of recurring fractures is also not the same.

In this study, it was concluded that combined spinal degenerative scoliosis is an independent risk factor for re-fracture after PKP surgery. Some studies believe that kyphosis or abnormal spine lines of force [17] changed the stress and weight-bearing state of the vertebral body, leading to re-fractures. This also proves from the side that scoliosis causes abnormal lines of force, which may be related to re-fracture. General data show that degenerative scoliosis of the spine is mostly concentrated in patients with 2 vertebral fractures (average 1.8 vertebrae). Such patients have different degrees of degenerative scoliosis of the spine. Combined with general data, from the perspective of the fracture-affected segments, re-fractures are concentrated in the T11–T12 or T12–T11, T12–L1, or L1–T12 segments, that is, the thoracolumbar vertebral body junction, where the stress concentration area is also a concentrated distribution area of degenerative scoliosis. Other re-fractures occurred at 1 or 2 or even 3 vertebrae separated from the original fractured vertebral body. From the survival analysis, it is further concluded that there is a significant difference between combined spine degenerative scoliosis and re-fracture. The median survival time of the combined scoliosis group is 48.98 months, which is significantly lower than that of the patients without scoliosis, which further indicates the combined spine degeneration Scoliosis is a high-risk factor for re-fracture after PKP. At present, most scholars believe that low BMD, fracture plane and the number of vertebral bodies, the amount of bone cement filling, the leakage of bone cement intervertebral space, the degree of compression of the fractured vertebral body, the postoperative height recovery, the degree of correction of the spine Cobb angle, etc. It may be related to the recurrence of vertebral fractures after PVP, so we included the above risk factors in the research category.

In theory, recurring vertebral fractures after PVP should be associated with BMD, and lower BMD may be a risk factor for recurring vertebral fractures after PVP [9]. When the BMD is lower, the adjacent segments of the fractured vertebral body are more prone to "column effect" and induce vertebral body fractures. Lee et al. [18] confirmed that low BMD is a high-risk factor for recurring vertebral fractures after PVP, and the lower the BMD value, the higher the risk of recurring vertebral fractures, which is similar to the results of this study. As an indicator of human health and fitness, whether BMI is a risk factor for recurring vertebral fractures after PVP has not yet been determined. Studies [19] have shown that BMI is correlated with osteoporotic fractures, and those with low BMI hip fractures are prone to occur, and those with high BMI are prone to vertebral compression fractures. Zhang et al. [20] meta-analysis results showed that low BMD and low BMI will increase the risk of recurring vertebral fractures after PVP; but there are also studies showing that there is no significant correlation between BMI and recurrence of vertebral body after PVP [21], which is similar to the results of this study. However, whether the recurrence of vertebral fractures after BMI and PVP is related still needs further research and a large number of accurate clinical controlled studies to confirm.

Whether the fracture plane and the number of initially fractured vertebrae are risk factors for recurring vertebral fractures after PVP is still a lot of controversies. The study of Yu et al. [10] confirmed that the plane of vertebral body fractures and the over-correction of the anterior edge of the fractured vertebral body are risk factors for recurring vertebral body fractures after PVP, especially the vertebral body fractures located in the thoracolumbar segment. There are also studies [22] where the risk of recurring vertebral fractures after surgery is correlated with the number of vertebral bodies in the initial operation; and the greater the number of vertebral bodies in initial compression fractures, the greater the impact on the biomechanics and pressure load of the entire spine after surgery. The greater the impact transmitted, this may increase the risk of recurring vertebral fractures. The follow-up results of this study showed that among the included observation indicators, the previous fracture history was one of the risk factors for recurring vertebral fractures after PVP. The risk of recurring vertebral fractures was 3.81 times higher than that of patients without a history of fractures. The above points are similar; however, the initial fracture number of the two groups of patients in this study did not find a significant correlation.

Bone cement leakage mainly includes extra vertebral space extravasation, paravertebral extravasation, and epidural extravasation, but most of them have no obvious clinical symptoms. As the most common complication of PVP surgery, most scholars currently believe that the leakage of the bone cement intervertebral space may be related to the re-fracture of the adjacent segment of the vertebral body after the operation. There is currently no uniform conclusion on the amount of bone cement injected during surgery. A high dose within a reasonable range can reduce the risk of vertebral fractures. However, the amount of bone cement filling is not the better. Seel et al. [23] showed that an appropriate amount of bone cement can increase the stiffness and strength of the fractured vertebral body, while excessive filling of bone cement can increase the pressure load of the adjacent vertebral body, which will cause subsequent fractures. However, Li et al. [24] followed up 230 cases of single-segment OVCF patients after surgery and found that patients with less bone cement filling had a higher risk of re-fracture after surgery. Lee et al. [25] followed up and observed 188 cases of OVCF patients after PVP and found that there was no significant correlation between bone cement leakage and re-fracture of the adjacent segment of the vertebral body after the operation, and the fracture plane (thoracolumbar) may be risk factors for recurring vertebral fractures after surgery. The univariate analysis results of this study showed that there was no significant correlation between the amount of bone cement filling and the recurrence of vertebral fractures after PVP.

In short, as the application of PKP becomes more and more popular, more and more patients will experience re-fractures. For patients with severe degenerative scoliosis, we must be alert to the risk of re-fracture and prevent and intervene in osteoporosis as soon as possible. Also, the research subjects are mainly outpatients and inpatients in our hospital. It is not a multi-center large sample study, the selection of cases is small, and many patients come from remote rural areas. There are many shortcomings and other related factors are not included in this study. In the research, the interrelationship between these factors needs to be further explored in future research.

## Conclusions

Combined scoliosis is an independent risk factor for re-fracture after OVCF vertebroplasty, and it is also a possible high-risk factor for re-fracture after OVCF.

## Data Availability

The datasets collected and analyzed during the current study are available from the corresponding author upon reasonable request.
